The article "English Research Learning and Functional Research Based on Constructivism Theory and Few-Shot Learning" was published in 2022. Journal: Comput Intell Neurosci.

# English Research Learning and Functional Research Based on Constructivism Theory and Few-Shot Learning

**DOI:** 10.1155/2022/3698802

**Published:** 2022-01-31

**Authors:** Chengyun Li

**Affiliations:** Zhengzhou ShengDa University, Zhengzhou, Henan 455000, China

## Abstract

Research-based learning is a comprehensive practical course that requires students to identify research topics from their study life and social life and acquires knowledge and applied knowledge through independent inquiry in a way similar to scientific research. Under the framework of CT (constructivism theory), through the study of English research-based learning and its functions, starting from few-shot learning, a college English teaching model based on the integration of network and research-based learning is constructed to explore the realization method of this model in the teaching process. UCSR-EW (user context-aware semantic-aware recommendation for English words) algorithm is used to generate English word recommendation, and the English word records are represented by the semantic model. Then, the acceptance of English words is measured according to the learning stage and English word records, and then, the similar users are matched, and finally, the intelligent recommendation of English words is realized. CC (confidence coefficient) is introduced into the pronunciation error correction algorithm to improve the traditional pronunciation error correction algorithm, so as to improve the error correction effect.

## 1. Introduction

Research-based learning is a concept opposite to receptive learning. It has many important functions, which are mainly manifested in helping to cultivate students' scientific inquiry ability, scientific spirit, independence and cooperation, social responsibility, innovative spirit, and innovative ability, helping to develop students' awareness and habits of exploration, helping to turn the learning process into a process of independent exploration, stimulating and enhancing learning motivation, and helping to cultivate students' sustainable development ability [1]. Therefore, as the inevitable trend of the current university curriculum reform, research-based learning has also become the focus of attention in the English teaching circle [2, 3]. More and more researchers are discussing the connotation of research-based learning and its application in English courses from theoretical and practical perspectives [4, 5].

CT (constructivism theory) is an important branch of cognitive learning theory, which is the result of psychologists' in-depth research on the cognitive law of the human learning process, and the further development of learning theory from behaviorism to cognitivism [6]. Because the learning environment required by CT is strongly supported by the latest information technology achievements, CT is increasingly combined with the teaching practice of teachers, thus becoming the guiding ideology of deepening teaching reform in schools at home and abroad [7, 8]. In order to meet the needs of modern quality education, middle school English curriculum standards have been revised several times, requiring middle school teachers to teach with brand-new teaching concepts, teaching methods, and means, take students as the center, pay attention to students' emotional factors, intelligence development, learning methods training and ability training, and teach them how to learn [9]. To achieve this goal, educators should provide a beneficial environment for students to help them create their own opinions independently or collectively [10]. The popularity of multimedia and network technology also makes the student-centered teaching structure have the material conditions for realization.

The importance of students' participation in research-based learning activities cannot be overstated. A multiperson activity is more likely to generate this type of participation. Building a learning society [11] necessitates multiperson activities, which are not only required by learning content. User information and English word learning records are collected and uploaded to the recommendation system, and a new recommendation method based on user similarity, as well as the recommendation system's model and process under the group intelligence perception mode, is explored and designed. Detection algorithms are created for various types of errors. Finally, various error detection algorithms detect the pronunciation to be processed separately, and corresponding corrective suggestions are provided for the incorrect pronunciation based on the results of the detection.

## 2. Related Work

The development of cognitive psychology and metacognition research provides rich theoretical knowledge for the study of learning strategies. Especially, cognitive psychology uses the viewpoint of information processing to explore the psychological mechanism within cognition, which makes it possible for human beings to explore their own implicit learning [12, 13]. Literature [14] divides learning strategies into macrostrategies and microstrategies. The former has a wider range of applications, involving more factors of emotion and motivation; the latter involves more special knowledge and skills, has a closer relationship with the cognitive execution process, and is easily influenced by education. In Literature [15], according to the theory of information processing and metacognition, it is proposed that learning strategies include cognitive strategies and metacognitive strategies. The former is the related method and technology for directly processing information, while the latter is the related method and technology for monitoring and mediating the information processing process. Literature [16] divides learning strategies into eight categories: retelling strategies of simple and complex learning tasks and finishing strategies for simple and complex learning tasks, simple and finishing organizational strategies, comprehensive adjustment strategies, and emotional strategies. Literature [17] puts forward the importance and necessity of learning strategy training in English learning. Literature [18] pointed out that research-based learning is a learning activity in which students, under the guidance of teachers, choose and determine topics for research from nature, society, and life, and actively acquire knowledge, apply knowledge, and solve problems during the research process. Literature [19] also gives two types of research-based learning: project research and project design. It is considered that objective knowledge structure is internalized into the cognitive structure through individual interaction with it. The interaction between learners and the environment involves two basic processes: “assimilation” and “hue”.

A recommendation system is a software tool and technology that suggests items to users based on their preferences. These recommendations cover a wide range of decision-making processes, including purchasing goods, listening to music, and reading online news [20]. Cinema recommendations are made to a virtual community of movie aficionados via e-mail and the Internet bibliography [21]. Bibliography literature [22] introduces eight attack strategies, which are mainly divided into four categories: basic attack, weak cognitive attack, nuclear attack, and informed attack. The challenges of modeling the simulated human score at the process and result levels are listed in literature [23], and it is noted that in the field of speech features and speech recognition, it is currently impossible to model the evaluation process comprehensively. Literature [24] evaluates the speaker's speech at the phoneme level, which has the benefits of accurately locating the speaker's pronunciation errors, evaluating the similarity between the speaker's speech and the target speech, and detecting systematic differences by comparing with a standard speech database. The user's voice data should be scored in segments at the phoneme level, and the overall score of this voice should be calculated by combining the scores of each phoneme, according to literature [25].

## 3. Research Method

### 3.1. English Research Study Based on CT

The key to English research study is students' activities. It is a tool of language communication, and any tool has one characteristic activity. If people want to learn a language, they must master the language through activities, learn to communicate, and achieve the purpose of communication through restricted and purposeful language activities. The development of research-based learning is mainly manifested in two aspects:

1. The model of research-based learning gives students full freedom, makes students truly become the main body of learning, fully demonstrates students' autonomy, and creates a good space for students' individual development
2. The evaluation of research-based learning is not to compare students horizontally but to make every student have a successful psychological experience through positive evaluation, and have enough self-confidence, so as to motivate every student to make new progress and achieve new success on the basis of the original, thus inspiring the internal needs and motives for improvement and improvement, and starting internal vitality and subjective initiative [5]

The teaching effect is determined by the design of the teaching model. In essence, research-based learning is a type of resource-based learning. In order to fully embody the characteristics of resource utilization learning, self-discovery learning, negotiation and cooperation learning, and practical and creative learning, the construction of a college English research-based learning mode in a network environment should take full advantage of the network platform's advantages, such as diversity, sharing, expansibility, and interactivity, and fully utilize the advantages of the network platform, such as diversity, sharing, expansibility, and interactivity. CT learning is emphasized as a process in which students actively construct meaning. In order to cultivate their autonomous, research-oriented, and cooperative learning abilities, students should actively explore, analyze, and discover the essence of things and their interrelationships using various methods, resources, and tools that are beneficial to the construction of meaning, from mastering little knowledge to constructing a complicated knowledge network.

CT teaching thought includes the following aspects: knowledge view, learning view, student view, evaluation view, the orientation and role of teachers and students, and learning environment (Figure 1).

Learning is always associated with a certain social and cultural background, that is, the “situation”. Learning in the actual situation can enable learners to assimilate and lead out the new knowledge that they have learned so as to endow the new knowledge with a certain meaning. If the original experience cannot assimilates the new knowledge, it will cause the process of “adaptation”, that is, the original cognitive structure will be reformed and reorganized. In a word, only by “assimilation” and “adaptation” can the meaning of new knowledge be constructed.

Whether it is the study of language knowledge such as phonetics, vocabulary, and grammar or the cultivation of basic skills such as listening, speaking, reading and writing, student-centered, aiming at how to guide students to learn and teach them to learn. Teachers should be good at creating situations, stimulating students' interest and motivation, setting appropriate learning tasks, creating lively and diverse activity environments, providing ample opportunities for practical language communication, allowing students to explore and solve problems by using their knowledge and original abilities, and also using language knowledge to communicate in activities to complete various tasks.

Combining the dominance and operability of classroom teaching, this study constructs a college English classroom teaching model based on the integration of network and research-based learning (Figure 2).

Research-based learning mode relying on network technology is subject-oriented, which changes the teaching process from traditional inheritance to inquiry. Students use the Internet to do a lot of online reading and online audio-visual, get “information input”, accumulate materials, and then refine their own views, transfer the perceived information to oral, form materials for oral expression, and provide “speaking” with the contents and ways of oral communication through logical transformation of thinking.

Teachers use the Internet to create real problem situations, guide students to discover and put forward problems that need to be explored, and generate a strong desire for research based on the teaching objectives, based on the content of teaching materials, and based on the principles of creativity, practicality, and novelty. Because the information on the computer network is linked by hypertext, it is easy for students to become disoriented, making teacher guidance crucial. The author primarily provides advice to students when they are debating a topic that is off-topic or disorderly.

However, affirming students' primary role in learning does not negate teachers' hegemony in the classroom. The essence of teaching is guidance, and the shift in teachers' roles is more focused on the promotion of educational concepts and the innovation of teaching strategies, which is to set new and higher standards for teaching and educating people in the new situation, rather than on the transfer of teaching and educating responsibilities and status. In essence, student-centered education requires teachers to create favorable conditions for students' development and fully recognizes teachers' dominant position.

Teachers should provide topic-related language materials, such as video or audio, while also supplementing literature materials with orientation and the appropriate degree to integrate language learning and consolidation into the application. The task's input materials primarily come from English resources on the Internet, which are directly from the front lines of application and have authentic, rich, and practical characteristics. Through research-based learning, students find, sort, and use them, resulting in language acquisition.

### 3.2. UCSR-EW Algorithm

UCSR-EW (user context-aware semantic-aware recommendation for English words) algorithm uses word vectors to represent words, considers the relationship between English words from the semantic point of view, and, on this basis, introduces the context information of users, matches the words that users are interested in, and realizes intelligent recommendation of English words.

Word recommendation algorithm introduces the semantic model based on English word browsing records to calculate interest similarity among users. The context similarity between users is calculated by using the context information of users, and then, user similarity is calculated according to interest similarity and context similarity; the neighbor of the target user is selected according to the user similarity; neighbors generate neighbor recommendation lists according to their English word records; finally, all neighbor recommendation lists are merged to generate the final recommendation result. The specific algorithm framework is shown in Figure 3.

UCSR-EW algorithm first uses the trained semantic model to calculate the semantic similarity of words and then constructs the feature vector of English word browsing records.

Formula (1) is used to calculate the similarity between feature vector *f*_*u*_ and feature vector *f*_*v*_, that is, the interest similarity of user *u*, *v*:

(1) $$\begin{array}{c} {\text{Sim}}_{\text{ic}}\left(u,v\right)=-\sqrt[{2}]{\frac{\sum_{i=1}^{k}{\left(f_{u}\right)}_{i}^{2}-{\left(f_{v}\right)}_{i}^{2}}{k}}. \end{array}$$

Feature vector *f*_*v*_ represents the semantic similarity of user *v* English word browsing records in user *u* word dimension, so the interest similarity of user *u*, *v* can be calculated by calculating the normalized Euclidean distance between feature vector *f*_*u*_ and feature vector *f*_*v*_.

The age and geographical location of the user are used as context information, and the learning stage of the user is described by the context information of the user. The contextual similarity Sim_sc_ of users will be calculated according to the age similarity Sim_age_ and the regional similarity Sim_location_, as shown in the following formula:

(2) $$\begin{array}{c} {\text{Sim}}_{\text{sc}}=\alpha \cdot {\text{Sim}}_{\text{age}}+\beta \cdot {\text{Sim}}_{\text{location}}. \end{array}$$

Among them, *α*, *β*, respectively, represent the weight of age similarity Sim_age_ and regional similarity Sim_location_ in the calculation process of user context similarity Sim_sc_, satisfying the condition *α*+*β*=1.

User-aware word semantic-aware recommendation algorithm is a recommendation method based on user similarity, which matches the neighborhood of the target user, and then generates recommendation results according to the neighbors of the target user (users in the neighborhood). User similarity Sim_user_ can be calculated according to interest similarity and user context similarity, as shown in following formula:

(3) $$\begin{array}{c} {\text{Sim}}_{\text{user}}=W_{\text{ic}}\cdot {\text{Sim}}_{\text{ic}}+W_{\text{sc}}\cdot {\text{Sim}}_{\text{sc}}, \end{array}$$

where *W*_ic_, *W*_sc_ represent the weights of interest similarity Sim_ic_ and user context similarity Sim_sc_, respectively.

After English words are duplicated and sorted, English words with large semantic similarity will always be ranked first, so that English words with small similarity but appearing in many neighbors' recommendation lists will never appear in the recommendation results. The word scoring model considering the frequency of English words is shown as follows:

(4) $$\begin{array}{c} \text{score}=D_{i}\cdot {\text{Sim}}_{\text{word}}\left(w_{i}\right), \end{array}$$

where *D*_*i*_ is the number of times the English word *w*_*i*_ appears in the neighbor recommendation list.

### 3.3. English Pronunciation Error Correction Algorithm

At present, the error correction evaluation of English pronunciation mainly focuses on the evaluation of acoustic characteristics, and the user's voice signal is cut into phoneme-level voice signals by forced alignment. Then, an evaluation score is obtained by calculating various similarities between the voice segments of each phoneme level and the standard phoneme acoustic model library.

This study develops a reasonable pronunciation error correction algorithm based on the above evaluation process and discusses and improves acoustic model training, phoneme segmentation, and similarity evaluation based on the characteristics of Chinese people speaking English. This study introduces the concept of CC (confidence coefficient), which calculates the confidence parameters such as likelihood ratio, likelihood ratio, and segment time to measure the similarity between this phoneme speech segment and the standard acoustic model, in order to correct users' pronunciation errors at the phoneme level and provide meaningful feedback information to users.

The pronunciation of this voice segment is the standard pronunciation. If the CC value of the observed sequence and the model of the standard phoneme is not within the range of the threshold value, the phoneme pronunciation of this speech segment is not standard, so as to further determine the wrong pronunciation of the user.

Assume that the phonetic sequence of word work is cut into three phoneme segments through a forced alignment network, corresponding to phoneme *W*, phoneme ER, and phoneme *K*, respectively. Let us take the phoneme ER as an example. First, let the observation sequence of the segmented ER be *O*_*t*_, and the corresponding standard phoneme model be *λ*_ER_.

The acoustic likelihood value of the frame corresponding to the standard phoneme model ER is defined as *l*_*i*_(*o*_*t*_) where

(5) $$\begin{array}{c} l_{i}\left(o_{t}\right)=P\left(o_{t}|\lambda_{\text{ER}}\right). \end{array}$$

The likelihood of the inverse model corresponding to the phoneme ER is

(6) $$\begin{array}{c} l_{i}\left(o_{t}\right)=P\left(o_{t}|\lambda_{\bar{\text{ER}}}\right), \end{array}$$

where $\lambda_{\bar{\text{ER}}}$ represents the inverse model of the phoneme ER.

Therefore, in the above formula, Ben multiplies the difference of ranking by the proportional difference of logarithmic probability, so that the reliability value of each phoneme will be influenced by ranking and logarithmic probability. The following is the set formula:

(7) $$\begin{array}{c} \text{Confc}={\text{PLLR}}_{\text{ER}}\left(o_{t}\right)*\text{Confc,} \end{array}$$

where Confc stands for the final CC.

The ratio of the number of phonemes whose error correction results are completely consistent with the expert labeling results to the total number of phonemes is known as the correct rate of phonemes. The algorithm's error correction rate is the ratio of the number of incorrect phonemes corrected by the algorithm to the total number of incorrect phonemes marked by all experts.

## 4. Results Analysis and Discussion

### 4.1. Analysis of English Word Recommendation Algorithm

In the process of research, using the method of group discussion, students are required to cooperate and help each other, which embodies the spirit of cooperation and mutual assistance among students. When the results are displayed between groups, they compete to show each other, hoping that their group is the best and the most perfect, which stimulates students' competitive consciousness. Pleasant cooperation and fair competition are two essential spirits for talent development today.

Students' ability to communicate correctly with pronunciation and intonation can only be cultivated in the real communication situation because changes in English stress, intonation, and rhythm are influenced by the actual communication environment and purpose. As a result, teachers should combine teaching materials to create language situations in which students can negotiate meanings and exchange emotions in communication and interaction, thereby assisting students in understanding the communicative function of pronunciation and intonation and forming an understanding of the English language. When speaking, students should be able to think clearly and express themselves using a variety of pronunciations and intonations.

The goal of the experiment of the word recommendation algorithm is to evaluate the word recommendation algorithm. The accuracy rate precision and recall are used to evaluate the effect of the recommendation algorithm. The higher the accuracy rate and recall rate, the better the recommendation effect.

The input of the UCSR-EW algorithm includes the user information file and English word record file. In addition, the algorithm also needs to input English word record length, English word number in the recommendation list, interest similarity weight *W*_*ic*_, age similarity weight *α*, and user similarity threshold *λ*.

The key to learning a language is to imitate it. When students first learn how to pronounce vowels and consonants, it is critical that they imitate the pronunciation and practice it repeatedly in order to become proficient and accurate at it. Listening to the English pronunciations of many British and American people and imitating their pronunciation and intonation can help students to improve their English language skills.

The optimal value shown in Figure 4 is for the experimental data itself. When the experimental data change, the size of the optimal value and the value of the parameters may not be as shown in the experimental results.

In order to verify the performance of the English word recommendation algorithm proposed in this study, a comparative experiment was designed, and experiments of UCAR (user context-aware recommendation algorithm) algorithm and EWSAR (English word semantic awareness recommendation) algorithm were carried out on the same experimental data.

Without considering the browsing records of English words, the contextual similarity of users is the similarity of users, while the recommended English words will depend on the browsing records of other users with similar age and small city distance and have nothing to do with the English words browsed by the target users.  Figure 5 shows the improved results of age similarity calculation, and Figure 6 shows the experimental results of the UCAR algorithm.

The communicative approach is helpful to improve students' communicative competence and enable them to learn to use correct and appropriate pronunciation and intonation. Teachers can provide students with various real communication situations and help students to correctly understand and choose the pronunciation and intonation suitable for the language environment, so as to achieve the purpose of communication.

Comparison of performance between UCSR-EW algorithm, UCAR algorithm, and EWSAR algorithm is shown in Figure 7, and UCSR-EW algorithm is superior to UCAR algorithm and EWSAR algorithm in performance.

It replaced indoctrination with grammar instruction as the mainline of English instruction, and it transformed knowledge-imparting classroom instruction into ability-cultivating classroom instruction, improving students' interest in learning, assisting them in developing better learning strategies, improving their comprehensive English ability, cultivating their innovative spirit and practical ability, and improving teaching quality.

Of course, the single use of any kind of teaching method in teaching is not easy to get the best teaching effect. Teaching is an art in itself. Only by guiding teaching with advanced educational concepts, taking the best teaching methods that meet the needs of the times, such as research-based learning as the leading factor, and combining all kinds of good teaching methods and creatively designing teaching can you get twice the result with half the effort.

The setting of learning objectives, the design of learning content, the provision of exercises, the transfer of adjacent knowledge, feedback, teaching assistance, learning evaluation, information organization, and other aspects should all well reflect the teaching nature. Teaching methods are not based on the learning content itself but attach importance to the creation of the learning environment. E-learning English does not just move the contents of English textbooks to the Internet intact but should combine learning theory and network characteristics to create a virtual learning environment for students and to pay attention to the organization of the teaching content, the richness, and the novelty of the content, so that students can find it worthwhile after browsing.

### 4.2. Analysis of Pronunciation Error Correction Algorithm

The main content of this section is to give the experimental results of adding the CC metric mentioned above to improve the traditional pronunciation error correction algorithm based on log likelihood. The experiment is designed and analyzed the experimental results in detail. The lower the threshold value, the more rigorous the algorithm is, the lower the phoneme accuracy rate, and the higher the threshold value, the looser the algorithm recognition, and the higher the phoneme accuracy rate.  Figure 8 shows the phoneme accuracy of the traditional log-likelihood ratio and improved CC-based error correction algorithm.

The CC-based error correction algorithm outperforms the traditional log-likelihood algorithm in terms of phoneme accuracy, as shown in Figure 8. It is necessary to identify correctly pronounced phonemes in order to provide reliable feedback to users, but it is not sufficient to do so alone. The scale of phoneme recognition is relaxed as the ranking domain value increases, and the algorithm's error correction rate decreases. Although the user's pronunciation is assumed to be the same as the standard phoneme, experts have determined that the user's pronunciation is incorrect. At this time, the system missed a detection error, lowering the system's error correction rate.

The following experiment is designed to discuss the relationship between the correct rate of phonemes and the error correction rate of the algorithm. The experimental results are shown in Figure 9.

From the above experiments, it can be seen that with the increase of the threshold value, the limitation of the algorithm on phoneme ranking is relaxed, and the phoneme accuracy rate increases, but the phonemes that users send wrong may also be regarded as correct phonemes, so the error correction rate of the system will decrease accordingly.

In this way, by using the sigmoid function, the CC value relative to each phoneme model is limited between [0,1].  Figure 10 shows a discussion about the constant port and the relationship between CC value and rank when *α* takes different values.

English research-based learning evaluation is a type of evaluation that aims to fulfill the full scope of the evaluation. It emphasizes that the core of evaluation is students' absorption and mastery in the learning process, emphasizes the role of evaluation in students' development, and pays attention to positive encouragement and encouragement. It takes the promotion of students' development as the fundamental purpose, takes the promotion of students' development as the orientation, embodies the people-oriented thought, emphasizes that the core of evaluation is students' absorption and mastery in the learning process, emphasizes the role of evaluation in students' development, and pays attention to positive encouragement and to students' own interpretations of various phenomena, listen to their current perspectives, consider the origins of these ideas, and assist students in expanding or revising their own explanations, pay attention to students' personal development, and do not dismiss external guidance, such as teacher influence, pay attention to student inspiration and induction during teaching activities, and guide students through discussion activities and connection reasoning to explore and find problems, solve problems, and acquire knowledge.

A colorful learning environment for students is created by creating situations that meet the requirements of teaching content and clues that suggest the relationship between old and new knowledge and help students to construct the meaning of what they are currently learning, to pay attention to the cultivation of cross-cultural awareness, method guidance, and strategy training, and to pay attention to guiding students to explore and discover the research-based learning style not only trains students' thinking but also cultivates their learning ability.

With the rapid development of multimedia computer and network education applications, CT is showing its strong vitality and expanding its influence in the world. Studying some learning theories of CT and carrying out teaching practice based on CT will carry out quality education with moral education as the core and cultivating students' spirit of exploration and innovation, active research and learning, cooperative learning, and practical ability as the focus, and promote the reform of teaching materials, which will have far-reaching influence and positive promotion.

## 5. Conclusion

Research-based learning is a teaching method in which subjects and objects are transformed and promoted by one another. This teaching model embodies the student-centered educational philosophy and emphasizes language acquisition and learning in the process and practice through the use of modern teaching methods. The central tenet of CT is that students are self-control knowledge builders. Teaching is primarily concerned with assisting students in improving their cognitive abilities. The UCSR-EW algorithm is proposed, which calculates an English word score based on semantic similarity and frequency of occurrence of English words and then recommends English words based on the score. In this study, we introduce CC into the phoneme error correction process and use it to calculate the CC rank of segmented phoneme segments and standard phoneme models to determine the accuracy of phoneme level in users' pronunciation. The results of the experiments show that including CC improves the correlation between system error correction and expert error correction significantly.

This study only looks at how phonemes are evaluated in spoken English, but there are many other aspects of spoken English that need to be highlighted for English learners, such as rhythm, and stress. Furthermore, the research and experiment in this study did not take into account the impact of regional dialects on English pronunciation. This will be the subject of more research in the future.

## Figures and Tables

**Figure 1:** Teaching thought of CT.

**Figure 2:** Web-based research-based learning model of college English.

**Figure 3:** English word recommendation algorithm framework.

**Figure 4:** Experimental result.

**Figure 5:** Improved results of age similarity calculation.

**Figure 6:** Experimental results of UCAR algorithm.

**Figure 7:** Algorithm performance comparison.

**Figure 8:** Comparison chart of phoneme accuracy before and after improvement.

**Figure 9:** Relationship between error correction rate and phoneme accuracy rate of the algorithm.

**Figure 10:** Relationship between *α* and rank rankings.

## Data Availability

The data used to support the findings of this study are included within the article.
